RETRACTED

# Gene Expression-Assisted Cancer Prediction Techniques

**DOI:** 10.1155/2021/4242646

**Published:** 2021-08-19

**Authors:** Tanima Thakur, Isha Batra, Monica Luthra, Shanmuganathan Vimal, Gaurav Dhiman, Arun Malik, Mohammad Shabaz

**Affiliations:** ^1^School of Computer Science and Engineering, Lovely Professional University, Jalandhar, India; ^2^Chandigarh University, Chandigarh, Punjab, India; ^3^Department of CSE, Ramco Institute of Technology, Rajapalayam, Tamil Nadu, India; ^4^Department of Computer Science, Government Bikram College of Commerce, Patiala, India; ^5^Arba Minch University, Arba Minch, Ethiopia; ^6^Chitkara University Institute of Engineering and Technology, Chitkara University, Punjab, India

## Abstract

Cancer is one of the deadliest diseases and with its growing number, its detection and treatment become essential. Researchers have developed various methods based on gene expression. Gene expression is a process that is used to convert deoxyribose nucleic acid (DNA) to ribose nucleic acid (RNA) and then RNA to protein. This protein serves so many purposes, such as creating cells, drugs for cancer, and even hybrid species. As genes carry genetic information from one generation to another, some gene deformity is also transferred to the next generation. Therefore, the deformity needs to be detected. There are many techniques available in the literature to predict cancerous and noncancerous genes from gene expression data. This is an important development from the point of diagnostics and giving a prognosis for the condition. This paper will present a review of some of those techniques from the literature; details about the various datasets on which these techniques are implemented and the advantages and disadvantages.

## 1. Introduction

DNA holds the genetic information of an organism for protein synthesis. The basic building block of DNA is called a nucleotide. It is made up of phosphate, deoxyribose, sugar, and four nitrate groups. These are generally inherited from parents to offspring, containing the genetic makeup required for the offspring to develop. The order in which these groups order themselves decides the traits of an organism, and this ordered arrangement is called a gene which is essential in protein synthesis. There are various types of DNA. A-DNA: DNA of this type is of right-handed double-helical type. DNA attains this configuration when short of moisture, dehydrated, or present in higher ionic concentrations. B-DNA: the standard format maintained by DNA during normal conditions in which life thrives, containing ten bases per rotation. C-DNA: complementary DNA is synthesized in a unique process called reverse transcription in the presence of a catalyst named transcriptase. D-DNA: it is an extremely rare configuration, and very little is known about it yet. Z-DNA: DNA of this type is of left-handed double-helical type. DNA attains this configuration when it is present in higher salt concentrations. It is similar to A-DNA but is left-handed in structure.

RETRACTED

RNA is a component that is primarily responsible for protein synthesis. It is helical in structure, single-stranded, and so it can easily fold upon itself to form other compounds. It is made up of phosphate, ribose, sugar, and four nitrogen bases. There are various types of RNA. tRNA, short for transfer RNA, is used to convert mRNA to protein. mRNA (messenger-RNA) takes information from DNA to the cytoplasm, where proteins are produced. rRNA, short for ribosomal RNA, is a part of ribosomes that synthesizes proteins that are further processed to form an essential protein. snRNA, short for small nuclear RNA, plays a pivot role in splicing introns and RNA processing [1].

“The process of transcribing a gene's DNA sequence into the RNA that serves as a template for protein production is known as gene expression” [2]. “Gene expression is the process by which the genetic code or the nucleotide sequence of a gene is used to direct protein synthesis and structure of a cell. Genes that code for amino acid sequences are known as structural genes.” Gene expression is usually carried out in two essential phases, namely, transcription and translation [3]. The process of translating the information encoded in a gene into an end gene product such as protein, rRNA, tRNA, or snRNA is known as gene expression. It is a sequence of the process mentioned above, like transcription and translation, which collects various subprocesses like initiation, translation, termination, and posttranslational processing. Gene expression is the basis for different life-developing processes where essential cells grow and develop their shape and specialized functions. It can be controlled to modify and obtain the desired functional proteins. Various other vital processes like adaptation to a specific environment, etc., are based upon this process. The significance of gene expression is rapidly increasing in various life sciences with the rise in technological standards. This analysis usually means the procedures to be undergone for spotting the target gene. It enables us to experiment with the various genes and traits they are responsible for in an organism. Some specific procedures in gene expression could allow us to create hybrid or mutated organisms. If cells of the same type are clubbed together, it will act like an organ [4].

### 1.1. Deep Learning

Deep learning (DL) is a subset of machine learning. DL has so many applications, such as detecting cancer, spotting in elephants, and developing games. The researchers are much interested in DL because of multiple reasons: the algorithms of DL provide promising results in solving complex problems, the data and the resources that are required to obtain the products are readily available, and many algorithms are coming into practice in a day-to-day world [5]. One kind of machine learning is deep learning. The machine learning algorithms are of two types: supervised and unsupervised. The deep learning algorithms depend on one of the optimization algorithms known as stochastic gradient descent. The machine learning algorithms work very well in different problems. However, these algorithms have not performed well in the main issues of AI, such as recognition of speech and recognition of objects. This problem acts as a motivator to the development of DL [6].

RETRACTED

Deep learning teaches computer systems to perform work in such a manner that comes so naturally to human beings: learn by illustration. It has become an essential technology behind driverless cars, causing them identifying a stop sign or discerning a pedestrian from a light pole. It acts as a secret for regulating sound in customer devices such as laptops, TVs, and hands-free devices. Deep learning is gaining a lot of attention. It is producing promising results which were impossible to obtain earlier. The system can learn directly from voice, text, and pictures for various classification jobs in deep learning.

There are so many deep learning applications in almost every industrial field, such as automatic driving and medical equipment. Some of the applications are defined as follows:

1. *Automated Driving*. The concepts of deep learning have been used by automotive developers to automatically identify artifacts like stop signs and traffic signals. This also employs deep learning to recognize pedestrians, which aids in the reduction of accidents.
2. *Aerospace and Defense*. DL has been used to classify objects that locate areas of concern from satellites and organize safe or unsafe areas for forces.
3. *Medical Research*. The researchers who are focused on classifying cancer cells are also using the methods of deep learning. The groups working at the University of California, Los Angeles (UCLA) have developed one microscope. The microscope has been trained using a high-dimensional dataset so that it can find the cancer cells accurately.
4. *Industrial Automation*. Deep learning also has its application in industrial automation. It is used to find the dangers associated with cumbersome and large machines.
5. *Electronics*. Various electronic devices that we use in our homes respond to our voices. All those devices work on the principle of deep learning [7].

RETRACTED

In this paper, gene expression data assisting various cancer prediction techniques have been presented. There are so many techniques from machine learning and deep learning that are available in the literature. However, our kind motive is to compare various existing methods to find a suitable process. The left-over part of the paper is partitioned as follows: Section 2 includes a description of various available techniques and a comparison table with information on multiple datasets.  Section 3 introduces the findings, and conclusion is in Section 4.

## 2. Related Work

We have reviewed various techniques for predicting cancer using the data of gene expression as discussed in Table 1. We have also presented one table with details regarding different methods, findings, and datasets various authors have used in their work.

In [8], Golub et al. have described a method based on gene expression to classify cancer, and DNA microarrays have also monitored the proposed method. It has been found that the described method to classify cancer is feasible and provides a way to predict classes of cancer without any prior knowledge. In [2], Slonim et al. have proposed a sample classification method for gene expression data based on computational analysis. The author also provides a way to use predictors to check the lifetime of new classes. The proposed approach offers a way for future work on molecular classification. In [9], Khan et al. proposed a framework dependent on Artificial Neural Networks (ANNs) for classifying cancers into specific groups. The method is based on signatures of gene expression. The proposed approach has been augmented using small round blue cell tumors (SRBCTs) model. With the help of this new method, all samples have been correctly classified and identified the genes. The proposed approach was put to the test with new models to see how well it worked.

In [10], Radmacher et al. have proposed one method for predicting the classes of predefined tumors based on gene expression profiles. The compound covariate prediction method has been used. The process is performing well, but still, there are some issues in the classification through the predictor. In [12], Pomeroy et al. have developed a method of classification based on DNA microarray gene expression data. It has been found using Principal Component Analysis (PCA) that medulloblastomas are molecularly different from other types of tumors. The proposed method also supports earlier findings regarding medulloblastomas that are derived from cerebellar granule cells. In [13], Weng et al. have facilitated this method to overcome one of the problems of supervised learning that is based on PCA and Fisher Analysis (FA). It has been found that the proposed method can also be used for gene expression analysis in supervised learning. It has been found that the data for gene expression in lung adenocarcinomas is also distributed in high-dimensional space and attributes are linearly discriminated.

RETRACTED

In [15], Duan et al. have presented a backward elimination procedure-based feature selection technique. The presented approach outperforms the original SVM-RFE method. It has also been found that several training partitions can be used as test sets for the gene expression-based cancer classification, as a performance quality metric. In [16], Berger et al. have presented a method that sets the variation patterns in 2 biological inputs, and Generalized Singular Value Decomposition (GSVD) acts as the base for it. It is found that the method is effective. The suggested approach is also applicable to a wide range of shared copy numbers and studies based on expression. In [17], Xu et al. have presented a method focused on semisupervised ellipsoid ARTMAP and PSO for separating tissues of a tumor with the help of analyzing the profile of gene expression. Compared to four other methods of machine learning, the approach outperformed them all on three other datasets, demonstrating that the classification accuracy variance is hugely significant. There are some problems related to noise and dimensionality.

In [18], Jung-Hsien Chiang and Shing-Hua Ho have introduced a prediction approach that uses a radial basis function NN and a rough-based method of feature selection. The method can be used to discover the unique features and defining centers close to the right ones. It has been found that this new method is having a high accuracy rate for classification. In [19], Zhiwen Yu and Hau-San Wong have presented a method for discovering classes of cancer from gene expression. It is found that Disagreement and Agreement Index (DAI) can be used to find the inner structure of all synthetic datasets and most of the cancer datasets. DAI also provides a higher validity index than other modernistic methods for gene expression.

In [22], Hou et al. have presented one approach based on genome-wide gene expression used to analyze a group of 91 patients. It has been discovered that the known gene signature can be used to classify non-small-cell lung cancer histopathologically. In [23], Salazar et al. have presented one method to predict cancer using gene expression. The main motive to create such a gene expression-based classifier is used to predict disease relapse at an early stage for patients suffering from colorectal cancer. ColoPrint significantly improves the predictive accuracy of pathological factors and MSI in patients suffering from stage II and III CRC. This also helps to identify stage II patients so that those can be safely treated without chemotherapy. In [24], Yuan et al. have proposed an integrative approach to learning a sparse DNA copy-number region interaction network with their corresponding transcription targets in breast cancer. It has been found that the proposed method produces a quantitative dependence score for copy numbers that differentiate cis- from trans-effects.

RETRACTED

In [26], Haseong Kim and Gelenbe have introduced a reverse engineering method based on the Bayesian Model Average that aims to combine all relevant gene interaction models. On a DREAM dataset created by nonlinearity stochastic processes, the presented method outperforms the other methods. It has been found that the proposed approach might be advantageous as it provides knowledge that is not extracted from traditional Differentially Expressed Genes (DEGs) methods.

In [27], Ashraf et al. have proposed a method for segmenting breast tumors based on multichannel Markov Random Fields (MRF). Multichannel MRF (area under curve—0.97) performs better than the single-channel MRF (area under curve—0.89) and performs better segmentation than other segmentation approaches such as structured segmentation cut algorithm.

In [28], Liao et al. have proposed a method based on supervised gene selection known as Locality Sensitive Laplacian Score (LSLS). The proposed approach was put to test on six datasets and it has been deduced that it is more accurate than other existing approaches.

In [29], Liu et al. have presented an approach for classifying samples of tumors from gene expression data based on robust PCA. The method has been tested on seven datasets, and it has been found that the procedure is accurate and feasible for the classification of tumors. In [30], Chen et al. have proposed D-GEX, one of the deep learning methods for inferring target gene expression from landmark gene expression. With a relative increase of 15.33 percent and a more minor error in 99.97 percent of the targeted genes, the proposed approach outperforms linear regression. The performance of this method has also been tested on the RNA-Seq-Based GTEx dataset. It has been found that it outperformed the technique of linear regression with a relative improvement of 6.57 percent and a more minor error in 81.31 percent of the targeted genes. In [31], Deng et al. have presented a fused network that identifies the stages of Kidney Renal Cell Carcinoma (KIRC). It combines the results of DNA methylation and gene expression. It has also been discovered that combining network-based functionality features from various types of data improves disease diagnosis.

RETRACTED

In [32], Chen et al. have identified the genes expressed in 32 normal tissues or cancer tissues used to investigate functional differences between genes widely and rarely expressed based on the overall gene expression results. The proposed approach aids in finding the landscape of gene expression and understanding how gene expression influences tissues and the cancer microenvironment. In [34], Elbashir et al., based on RNA-Seq gene expression results, have presented a lightweight CNN Breast cancer classification method. The proposed approach has been found to outperform other state-of-the-art techniques with an accuracy of 98.76 percent.

In [35], Khalifa et al. have developed a diagnostic method based on BPSO-DT and CNN for cancer using RNA-sequence gene expression data. The suggested method achieves the testing accuracy of 96.90 percent and outperforms the other related techniques. The technique is less complex as well as less time-consuming. In [36], Chun-Hou Zheng et al. have presented a robust method based on nonnegative matrix factorization (NMF) or sparse NMF to classify tumors from gene expression data. It has been found that it is very efficient and effective to classify tumors and normal tissues.

In [38], Wang et al. have developed an approach based on Dual Hypergraph Regularized PCA (DHPCA) to bicluster tumor gene expression data. It has been deduced that this is an excellent tool for biclustering. It has also been found that the method exposes those gene clusters which are having the same biological functions. There is one drawback of the method that it has not been evaluated thoroughly. In [39], Wang et al. have presented a model known as LGEPM that is used to extract the nonlinear features that affect gene expression. It has been found that the problem that occurred with the Library of Integrated Network-Based Cellular Signatures (LINCS) program has been solved by using this new method.

In [40], Khorshed et al. have proposed a multilayer framework based on CNN known as GeneeXpression Network (GeneXNet). It is used to classify the multitissues of cancer. To support the use of deep learning for biological use, a visualization of the proposed model has been presented with an accuracy of 98.9 percent. In [41], Ji et al. have turned to a gene selection method based on Partial Least Squares (PLS) to identify genes from high-dimensional data for the timely cure of cancer. It has been found that the method is efficient and robust. It provides good classification results in multicategory datasets also. In [42], Fang-Han Hsu et al. have proposed a single transcription model (ST) based on the Laplace–Stieltjes transform and numerical analysis. With the help of this method, the transcription factors (TFs) are uploaded after the specification of transcription. Mathematical models and simulations are used to evaluate functional disorders due to copy number alterations (CNAs). However, this could not be achieved using the Unlimited Transcription model (UT).

RETRACTED

In [43], Farouq et al. facilitated gene expression profiling in non-small-cell lung cancer (NSCLC). It leads to a better definition of NSCLC-related genes by reducing uncertainty and increasing decision reliability and validity. In [44], Kiranyaz et al. have presented a review on 1D convolutional NN, its applications, and comparison with 2D Convolutional Neural Network. It has also been found that 1D CNN requires less effort for training, and it is less complex since it works on small data. 1D CNN only works for low computational devices such as mobile and hand-held devices. However, on the other hand, if a large dataset is there and complex computations have to be done, the 2D CNN must be used. It has also been found that the more the parameters, the more the features to be extracted that make 2D CNN better than 1D CNN for large datasets. In [45], Wu et al. have proposed a 2D CNN method for the classification of images of ECG signals into normal and abnormal. The proposed method provides 98% accuracy. It has also been found that 2D CNN outperforms 1D CNN. 2D CNN method is precise and sturdy than 1D CNN.

## 3. Research Findings

In the light of the literature survey, it has been found that the gene expression data provides some added details that help to enhance the classification and diagnosis of cancer. Therefore, one can work with the gene expression data for better results. According to the work done in [35], the authors used BPSO-DT and CNN for differentiating cancer. They used five layers of NN architecture on a limited dataset of 2086 samples. However, there is also a multilayer CNN architecture available that can be used to achieve better accuracy [34, 35] and [40]. From [36, 38–42], it has been found that the algorithms used are machine learning algorithms as the dataset is more petite. However, if big data would be there, these algorithms will create a problem of overfitting to the training dataset. Therefore, we can use better algorithms to get better results. We can also use the large dataset and proposed techniques to achieve better performance on the relevant features [35].

Figure 1 compares some of the techniques from the literature used to predict cancer from the gene expression dataset. Convolutional Neural Network (CNN) has been used many times, and it provides good results with better accuracy than the other mentioned techniques.

RETRACTED

From [44, 45], it has been found that 1D CNN works where there is a small amount of training data and low cost implementation is required. In such situations, 2D CNN does not work due to the shortage of training data. It has also been found that 1D CNN requires less effort for training and it is less complex due to the fact that it works on small data. 1D CNN only works for low computational devices such as mobile and hand-held devices. However, on the other hand, if large dataset is there and complex computations have to be done, then 2D CNN must be used. It has also been found that the applications of 1D CNN use less hidden layers having less parameters (approx. less than 10 K), whereas on the other hand, 2D CNN has more layers with parameters more than 10 M. It means more parameters, more features to be extracted that make 2D CNN better than 1D CNN for large datasets.

From the literature survey, it has also been highlighted that CNN works very well for the images because of the hierarchical nature of the convolution layer. Convolution layer is the most important block of CNN architecture. The first hidden layer focuses on low-level features, then the second hidden layer on high-level features, and so on. Consecutive layers in CNN are not fully connected with each other and even it uses its weights again and again. It has less parameters than fully connected networks. There are some advantages of the CNN over other fully connected networks such as it takes less training time, less training data, and less risk of the problem of overfitting. CNN can detect the same feature at multiple locations when its kernel learns that feature. Images consist of various iterative features. This makes CNN good for working with images with lesser training data, and the high-dimensional features can be extracted. Large-size filters are used in 1D CNN. It means if a filter of size 7 is used, it would have only 7 feature vectors. However, in the case of 2D CNN, if a filter of size 7 is used, it would have 49 feature vectors. This is the reason 2D CNN provides high-dimensional features compared to 1D CNN [46].

## 4. Conclusion and Future Scope

Cancer is badly affecting a large set of population. If it is not diagnosed on time, it becomes difficult for the doctor to save the patient's life. There are many methods available in the literature to predict cancer. However, presently, gene expression data is attracting people towards it. As there is big data, various deep learning methods are used to predict the cancerous and noncancerous genes. Each technique has its pros and cons. The paper shows a review of some of those methods. From the study, it has been found that the gene expression data provides some added details that help to enhance the classification and diagnosis of cancer. Therefore, it means one can work with the gene expression data for better results. It has also been found that machine learning algorithms are used when the dataset is petite. However, if big data would be there, these algorithms will create a problem of overfitting to the training dataset. Therefore, we can use deep learning methods to avoid these problems.

RETRACTED

## Figures and Tables

**Figure 1:** Comparison of various prediction techniques.

**Table 1:** Review of various cancer prediction techniques.

Sr. no.	Paper name	Objective	Technique/tool	Dataset	Findings
1	[8]	To design a method to classify and predict classes of cancer	Neighborhood analysis, DNA microarrays, self organizing maps	27 ALL samples from Dana-Farber Cancer Institute, 11 adult AML samples from the Cancer and Leukemia Group B (CALGB) leukemia cell bank	Feasible method. Proper experimental care is required

2	[2]	To classify samples of cancer for gene expression data	Computational analysis, affymetrix oligonucleaotide arrays, neighborhood analysis, genecluster software	38 leukemia samples (11 AML, 27 ALL), for testing 34 samples (14 AML, 20 ALL)	Genes with no correlation provide a better result, and the median prediction strength is 0.86

3	[9]	To specify the specific categories of cancer using their gene expression	ANNs, cDNA microarrays, DeArray software	NCI, ATCC, MSKCC, CHTN, DZNSG, National Institutes of Health	It can work with nonlinear features also. It is robust. It also achieves high sensitivity and specificity.

4	[10]	To create a framework for predicting predefined classes of tumor	Compound covariate prediction, BRB ArrayTools	Hereditary breast cancer dataset of 22 patients [11]	Good setter for comparing prediction methods. Require some improvements.

5	[12]	To develop a classification system for DNA microarray gene expression data	SOMs, Cluster and TreeView software, PCA, KNN	Multiple datasets have been used, such as one with 99 samples, the other with 42 selections,	Gene expressions provide an excellent way of diagnosing patients with medulloblastomas

6	[13]	To propose a method that performs classification on interval-scaled attributes basis	PCA, FA, fuzzy FA	203 samples (a subset of the actual dataset used in [14])	Successfully used in supervised learning. FA provides more information compared to surgical-pathological staging

7	[15]	To propose a method for gene feature selection	Multiple SVM-RFE	Four gene expression datasets available on Kent Ridge Bio-Medical Data Set Repository	MSVM-RFE has classification accuracy better than SVM-RFE. SVM's performance has been improved.

8	[16]	To propose a framework for addressing the problem of integration of different data types	Generalized singular value decomposition	Fourteen breast cancer cell lines from American Type Culture Collection	Gene expression and copy number data are being analyzed. Improvements can be made to use other data types also.

9	[17]	To propose a method used to find tissues of the tumor with different gene expression data	ssEAM, PSO	NC160, acute leukemia, ALL dataset	ssEAM performs better than PNN, ANN, LVQ1and KNN at a 0.05 significance level

10	[18]	To present a selection method for analyzing gene expression data	RBF neural network, rough based feature selection method, naïve Bayes, linear SVM	ALL, AML, lung cancer and prostate cancer dataset (http://sdmc.lit.org.sg/GEDatasets/Datasets.)	The best classification accuracy rate of 99.8%

11	[19]	To present a framework for discovering cancer classes.	Permutation technique, cluster ensemble, cluster validity index (DAI)	3 synthetic and 4 real datasets (leukemia [2], Novartis multitissue [20], lung cancer [14], St. Jude [21])	DAI finds the number of classes correctly and outperforms other existing methods

12	[22]	To present a method based on gene expression for classifying NSCLC	Hierarchical clustering, SpotFire decision site, proportional hazards model	91 NSCLC, six normal lung tissues from GSE3526 (Duke University)	Gene signatures provide the best way for histopathological classification

13	[23]	To propose a classifier predicting disease in CRC patients	Agilent 44K oligonucleotide arrays, Kaplan–Meier method, unsupervised hierarchical clustering	188 training samples (NCI, LUMC, SGH) and 206 testing samples (Institute Catalad'Oncologia, Spain)	Eighty-six percent of patients of the validation dataset are identified as low-risk patients. First prognostic technique for CRC

14	[24]	To propose a framework that combines genome-wide copy number and expression data	L_1_-L_2_ constrained regression, local and global search strategies	89 samples of breast cancer Dataset (UG San Francisco and California Pacific Medical Center [25])	Outperforms other existing methods accuracy

15	[26]	To propose a framework that combines other models that describes gene interaction.	Bayesian model, Gibbs distribution, ANOVA test, parallel programming with GPU/CPU	GSE4290, DREAM dataset	Specificity of 0.99 has been achieved. Better performance than Enet and VAR

16	[27]	To propose the extended framework for segmentation of breast tumor	Multichannel MRFs, kinetic observation model, Gaussian mixture model	DCE MRI images of breast cancer	AOC of 0.9 has been achieved using multichannel MRF compared to AOC of 0.89 in single-channel MRF. Better segmentation results when applied to SVM

17	[28]	To propose a gene selection method	LSLS, wrapper method, SVM	Six datasets available at Kent Ridge Biomedical Data repository	LSLS performs better than KW and SPFS

18	[29]	To present a novel method classifying tumor samples.	RPCA, LDA, SVM	Nine different publically available datasets (acute leukemia data [2], colon cancer data, glimos data, medulloblastoma data, prostate cancer data, 11_tumor data, and brain tumor data)	Performance is measured using LOO-CV, accuracy, and AUC. A feasible and effective method.

19	[30]	To propose a method based on deep learning for inferring target genes expression	D-GEX	Microarray GEO dataset, RNA-Seq-based GTEx dataset	Outperforms linear regression (15.33 relative improvement) and KNN. The lower error rate in most of the genes (81.31%).

20	[31]	To develop a fused network identifying KIRC stages	Gene expression and DNA methylation data, SNF, SNFTool, sparse partial least square regression, LASSO label prediction method	The Cancer Genome Atlas KIRC data (TCGA data portal)	High prediction accuracy than KNN, MLW, and WDC. It is robust.

21	[32]	To classify widely and rarely expressed genes	Incremental feature selection method, mRMR, RNN	Gene expression dataset available at the Human Protein Atlas [33]	GO terms and KEGG are used at the functional level. Youden's indexes are 0.739 and 0.639 for normal and cancer tissues, respectively.

22	[34]	To develop a light-weight CNN for classifying breast cancer	CNN, array-array intensity correlation, R-Studio, batch normalization	Breast cancer dataset from Pan-Cancer Atlas	Achieves 98.76% accuracy

23	[35]	To propose a method for classifying different types of cancer.	BPSO-DT, CNN, deep learning	Cancer types: RNA sequencing values from tumor samples/tissues available at Mendeley datasets	It achieves an accuracy of 96.90%. Various evaluation parameters are recall, precision, and F1 score.

24	[36]	To propose a method based on NMF to classify tumor	NMF, SNMF, SVM	Colon cancer dataset [37], acute leukemia dataset, medulloblastoma dataset	It is effective and efficient. The effect of sparseness is low.

25	[38]	To propose a model for biclustering data of gene expression.	PCA, GLPCA, DHPCA,	SRBCT, medulloblastoma, colon cancer, 11_Tumors	It is compared with PCA, GLPCA, GNMF, ONMTF, and NMTFCoS. It provides better accuracy than others.

26	[39]	To present a framework for predicting the expression of genes employing nonlinear features	Unsupervised clustering algorithm, L-GEPM, LSTM neural network	GEO data from LINCS cloud, GTEx, and 1000G RNA-Seq data	Performs better than D-GM, LR-L1, and KNN-R. Target genes extracted are much closer to the actual gene expression. Flexible and superior for NL features.

27	[40]	To propose a multilayer framework to classify multitissues of cancer.	CNN, RNA sequencing, supervised learning, stochastic gradient descent optimization, back-propagation	11093 samples from the Cancer Genome Atlas	98.93 percent overall accuracy and 0.99 AUC have been achieved

28	[41]	To propose a gene selection method that can classify tissues in multicategory datasets	PLS, linear support vector classifier, MATLAB, OSU_SVM3.00 toolbox linear SVC, SVM	MIT AML and ALL dataset, SRBCT datasets	It is efficient and robust. It works well for both two-category and multicategory datasets.

29	[42]	To propose an ST model for finding the effects of CNAs	LST and NA, dynamic modeling, transcriptional bursting, transcriptional oscillation, circular binary segmentation	NCBI/GEO database	It shows the use of mathematical theory to investigate the findings and for a better understanding of cancer bio

30	[43]	To propose a muti-fusion-based method for profiling gene expression under nonthermal plasma treatment.	Dempster–Shafer method, fuzzy C-Means clustering method, MATLAB R2016b	NCBI Gene Expression Omnibus under GEO (GSE59997)	Reduces uncertainty and increases reliability. The use of C-means finds changes in genes in various nonthermal plasma treatments.

31	[44]	To present a survey of 1D CNN and its applications.	NA	NA	1D CNN works well with small data and where fewer computations are required. It also works where low-cost implementation is needed.

32	[45]	To propose a classification method for ECG signal images based on 2D CC.	CNN, Intel17-5930K CPU, and NVIDIA GTX1080 GPU	MIT-BIH Arrhythmia database	2D CNN outperforms 1D CNN. 2D CNN is more accurate and robust. 1D CNN works well with limited data.

RETRACTED

## Data Availability

Data will be made available upon request.
